The article "Big Data Technology Oriented to Wetland Resource Ecosystem Value Evaluation" was published in 2022. Journal: Comput Intell Neurosci.

# Big Data Technology Oriented to Wetland Resource Ecosystem Value Evaluation

**DOI:** 10.1155/2022/6815102

**Published:** 2022-05-30

**Authors:** Lifang Fan

**Affiliations:** ^1^School of Resources and Environmental Science, Hubei University, Wuhan 430062, China; ^2^Hubei Key Laboratory of Regional Development and Environmental Response, Hubei University, Wuhan, Hubei 430062, China

## Abstract

In order to study a big data technology research for the evaluation of wetland resource ecosystem value. This paper proposes a wetland dimension oriented to the evaluation of wetland ecosystem services space attribute through big data coupling analysis framework. The framework used China's coastal wetlands as a case for empirical research and summarized the future direction of the research on the value evaluation of wetland ecosystem services in the era of big data. The result shows: Wetland Ecosystem Observation Network can obtain long-term series of dynamic data, remote sensing Earth observation can realize the integrated observation of space, space, and Earth, the combination of the two will help to build a wetland ecological big data observation system. The service value of China's coastal wetland ecosystem is 5010.32 × 108 yuan. The research results can effectively solve the problem of geographical heterogeneity and have reference value for the protection and management of the wetland ecosystem.

## 1. Introduction

With the rapid development of information technology, information acquisition methods and data analysis methods are undergoing drastic changes, data science, dominated by big data, has become the focus of attention in the academic world. Compared with traditional data analysis methods, big data is a new way of thinking, rely on comprehensive data to systematically solve complex scientific problems [1]. In terms of ecology, many scholars have also discovered the importance of big data and carried out related research, which provided new ideas for the scientific solution of many ecological problems. The formation mechanism of wetland ecosystem services is complex, the driving factors are diverse, due to natural interference, human activities, hydrological changes, vegetation succession, and historical differences in the development of specific areas, and wetland ecosystem services show significant temporal and spatial specificity and comprehensive characteristics. In the era of big data science, use of massive, high-dimensional, and variable wetland observation of big data to systematically study the value of wetland ecosystem services, and explore the big data comprehensive evaluation method of wetland ecosystem service value, it is an important breakthrough to achieve accurate assessment of the value of wetland ecosystem services [2]. The evaluation of the service function value of the wetland ecosystem is the basis for the protection and rational use of the wetland. Through the process of wetland evaluation, we can accurately understand the wetland and the various functions it provides for human beings and to make a reasonable quantitative evaluation on this basis, and also it is very important for wetland protection and reasonable and effective management of wetland [3]. Wetland ecosystem services, functions, and evaluation research began in the early twentieth century. In the early scholars' evaluation research on wetland ecosystem services, it is mainly done through the establishment of an indicator system or the use of questionnaires to evaluate the value of wetland ecosystem services to convert the value of ecosystem services into monetary value [4]. In the study of the service value of farmland ecosystems, Sahoo and Bhaskaran calculated the value of farmland ecosystem services based on the inflow of water from the river, and recommended to distribute the incoming water volume during the year, and stated that water rights trading, ecological compensation, multiple means to ensure the river ecological base flow were important [5]. Fu et al. constructed an economic analysis framework of land use transfer based on the theory of maximum utility and argued that in the context of ecological restoration of projects and urban expansion, the impact mechanism of cultivated land transfer in Shaanxi Province on the value of ecosystem services is of relevance [6]. Burlakova et al. combined Constanza's results after field research in China; it is believed that directly introducing foreign results into China can easily overlook the value of certain ecosystems. From this, a new unit price system for evaluating the value of ecosystem services in China is proposed [7]. Based on this, this paper proposes a wetland dimensional-spatial-attribute coupling big data analysis framework for wetland ecosystem service value assessment. This framework selected China's coastal wetlands as a case for empirical research and summarized the future direction of wetland ecosystem service function evaluation research in the era of big data.

The article "Big Data Technology Oriented to Wetland Resource Ecosystem Value Evaluation" was published in 2022. Journal: Comput Intell Neurosci.

## 2. Wetland Ecosystem

### 2.1. The Big Data Observation System of Wetland Ecosystem

Wetland ecosystem observation is to observe the ecological indicators of wetland regularly, the process of quantitatively acquiring wetland ecological quality and its change information. In terms of observation methods, wetland big data observations face various types of problems, complex structure, wide distribution, numerous elements, a series of issues such as dynamic changes. A comprehensive and scientific wetland observations require comprehensive use of modern technology to carry out a full indicator system, time continuous, spatial continuous, multi-scale joint, and other systematic observations. In terms of technical means, a complete wetland field observation network needs to be established. For wetland big data observation, establish a scientific and practical wetland observation index system, make full use of new remote sensing observation methods to strengthen the construction of a technical system for the acquisition, transmission, storage, and management of wetland big data [8].

### 2.2. Big Data of Wetland Ecosystem Observation Station Network

China has a vast territory and different types of landforms. The geographical environment is complex and the climatic conditions are diverse, and it is one of the countries in the world with complete types and abundant numbers of wetlands. According to the classification of wetland types in the “Wetland Convention”, there are 31 types of natural wetlands and 9 types of constructed wetlands in China. The main types of wetlands include marsh wetlands, lake wetlands, river wetlands, estuary wetlands, natural and constructed wetlands such as coastal tidal flats, shallow waters, reservoirs, ponds, and rice fields. The types of wetlands are diverse and widely distributed so that the observation of wetlands must also be based on types of wetlands and the distribution of wetlands. The importance of wetlands are carried out purposefully at multi-level observations from key wetlands to general wetlands, network observation system from inland to coastal, and from inland freshwater wetlands to inland saltwater wetlands [9]. The wetland ecological station establishes long-term observation points and observation sample plots in important and typical wet areas. Long-term positioning observation of the ecological characteristics, ecological functions, and human disturbance of the wetland ecosystem, in order to reveal the mechanism and regulation methods of the occurrence, development, and succession of wetland ecosystems to provide scientific basis for protection, restoration, reconstruction, and rational use of wetlands. The establishment of the wetland ecological station provides a good technical platform for observing the wetland ecosystem, and it is an important guarantee for wetland research and scientific development of wetland.

### 2.3. Wetland Ecosystem Service Value Evaluation Based on Big Data

Supported by the big data of wetland ecosystem observation, study the applicable ecosystem service big data mining and coupling analysis method system. It is the key to realize the service value assessment of wetland ecosystem. Ecosystem observation big data has the characteristics of massive data, complex dimensions, and numerous variables, bringing unprecedented difficulties to data mining and analysis. For this reason, based on the theory of wetland ecosystem service value evaluation, the general research paradigm is defined as follows:

(1) $$\begin{array}{c} Y=\left[X\right]\left[S\right]\left[C\right]. \end{array}$$

In the formula, *Y* is the dependent variable, refers to the ecosystem service functions provided by wetlands, generally multidimensional service function; *X*, *S* and *C* are independent variables, respectively, referring to the quantitative and qualitative representations of the service value of wetland ecosystems, where *X* is the representative quantity of wetland resource information. Generally it is the spatial data of wetland distribution, *S* is the qualitative ecological parameter information, generally it is wetland attribute data. *C* is the evaluation method system of wetland ecosystem service value, generally standardize different service evaluation methods, by coupling comprehensive wetland observation data, and construct a data-driven wetland ecosystem service value evaluation method [10]. Based on this, decompose the big data research system of wetland ecosystem service value evaluation into dimensional analysis methods, spatial analysis methods, attribute analysis methods, and comprehensive coupling methods.

The article "Big Data Technology Oriented to Wetland Resource Ecosystem Value Evaluation" was published in 2022. Journal: Comput Intell Neurosci.

#### 2.3.1. Space Analysis

Spatial analysis is a quantitative characterization of wetland resource conditions and services provided from the perspective of wetland spatial distribution. The spatial expression can use quantitative data such as the spatial distribution of wetlands, the distribution of wetlands, and the geographical weight matrix of wetlands. The analysis unit can use geographic grid, geomorphological unit [11], land unit, wetland unit, and other methods, and the analysis method can adopt the form of spatial correlation matrix. The relationship between land types and ecosystem service types and their ability to provide corresponding services are represented by a supply matrix. The conversion matrix is listed in Table 1 The type of land indicated in the row of the table and the type of service indicated in the column are the wetland types and ecosystem services of the target wetland, *N* provides the relative weight of the ecosystem service capability of the column for the land type of the row, and it is obtained through dimensional analysis and conversion, and finally normalized to an integer value between 0 and 10, as the standard capability of this land type to provide wetland ecosystem services [12].

The article "Big Data Technology Oriented to Wetland Resource Ecosystem Value Evaluation" was published in 2022. Journal: Comput Intell Neurosci.

Attribute indicators are generally divided into three categories: natural indicators, environmental indicators, and socioeconomic indicators: (1) Natural indicators mainly refer to the natural characteristics of wetlands, which are the internal factors of the service supply capacity of wetland ecosystems. (2) Environmental indicators mainly refer to the natural environmental information where the wetland is located, and are the objective factors that mainly affect the service supply capacity of the ecosystem. (3) Socioeconomic indicators mainly refer to the socioeconomic information where the wetland is located [13], and it is an objective factor that mainly affects the value of ecosystem services. Commonly used natural, environmental, and socioeconomic indicators are listed in Table 2.

### 2.4. Big Data Coupling for Wetland Service Value Evaluation

On the basis of the general research paradigm of wetland ecosystem service value evaluation, a logarithmic model of dimensionality-space-attribute big data coupling model is proposed to realize the integrated analysis of big data of wetland ecosystem service dimensions, space, and attributes. The dependent variable of the model is the total value of wetland ecosystem services, and the independent variables are wetland type, supply matrix, wetland natural, social, economic index vectors, etc. [14]. The expression of the model is

(2) $$\begin{array}{c} InV_{ij}=\beta_{0}+\beta_{w}\beta_{w}X_{wj}+\beta_{c}X_{di}X_{cj}+\beta_{m}X_{mi}+U_{ij}. \end{array}$$

In the formula, the dependent variable *InV*_*ij*_ is the value of the *i*-th wetland ecosystem evaluation in the *j*-th wetland (yuan/(hm2·year)); *X*_*w*_ is the natural vector of wetland, and mainly refers to wetland scale, wetland type, and wetland ecosystem service function, etc.. *X*_*c*_ is the wetland environment vector, including GDP, industry type, population density of the city, where the wetland is located. *X*_*d*_ is the total value of all ecosystem service benefits of the wetland, the calculation method is *X*_*d*_=∑*N*_*ij*_*A*_*ij*_, where *A*_*ij*_ is the area of type *i* wetland, *N*_*ij*_ is the standard capacity value of the *j*-th ecosystem service corresponding to the *i*-th wetland category, see wetland category and wetland ecosystem service supply matrix. *X*_*m*_ is the vector of the evaluation technique, constants for the evaluation methods of various services. The subscripts *i* and *j* indicate the *i* evaluation in the *j* study. *β*_0_ is a constant, *β*_*w*_, *β*_*m*_, *β*_*c*_ are the regression coefficients in their respective group variables including explanatory factors; *U* is the error term [15].

The article "Big Data Technology Oriented to Wetland Resource Ecosystem Value Evaluation" was published in 2022. Journal: Comput Intell Neurosci.

### 2.5. Evaluation Method of Wetland Ecosystem Service Value

The direct market value method is to use the fair price in the active trading market to evaluate through the direct market method. The market price method is simple and practical, and its value expression is intuitive and easy to understand. It is mainly used in ecosystems that can produce direct material by-products, such as animal and plant products, shipping value, and water supply. However, this method can only measure the direct benefits of the material output and service functions of ecological assets, ignoring its indirect benefits, and it is easy to underestimate the overall value of ecological assets. Through the direct market value method, its value expression form is similar to that of ordinary assets, and the price expression form is intuitive and clear. It belongs to the personal or national wealth in the usual sense and is a biological resource in the general concept. To a certain extent, ecological assets serve the functional value. The calculation method is as follows:

(3) $$\begin{array}{c} V=\sum \left(Si\times Yi\times Pi\right). \end{array}$$

In the formula, *V* is the direct use value, *Si* is the production area of the *i*-type material, *Y* is the unit yield *P* of the *i*-type material; is the market price of the *i*-type material.

Indirect market evaluation method. The main difference between ecosystem service value assessment and ordinary asset assessment is that ecosystem services have no direct material output, lack an active public trading market, and their value expressions are concealed, so conventional asset assessments such as market methods, income methods, and cost methods cannot be used. For example, the value of wetland water conservation, the value of flood control and storage, can only be evaluated by indirect markets such as construction costs assuming the same service function or economic loss caused by the lack of a certain ecological service change. The expression formula for this method is

(4) $$\begin{array}{c} V=U\\ =\sum Xi. \end{array}$$

In the formula, *V* is the value of the ecological service function; *U* is the price of the shadow project of the ecological service function; *Xi* is the cost of the *i*-th project in the shadow project.

The value equivalence table can dynamically evaluate the value of 14 major ecosystems and 11 types of ecological service functions. In different regions, adjustments are made based on the local basic farmland biomass factor of the research object, such as the formula:

(5) $$\begin{array}{c} \text{ESV}=\sum \left(S_{i}\times VC_{i}\right),\\ {\text{ESV}}_{j}=\sum \left(S_{i}\times VC_{ji}\right). \end{array}$$

The service function of regulating runoff refers to the function of wetlands as a reservoir, storing excess precipitation in rainy seasons, alleviating urban waterlogging, providing water sources in dry seasons, and alleviating the impact of droughts. For the functional value of runoff regulation, it is difficult to measure the benefits directly. Shadow engineering estimates the value of replacement runoff regulation that would otherwise be expended to make up for this function. The shadow engineering method refers to the construction of a new project to completely replace the service function that needs to be evaluated, and the value of a service function is replaced by estimating the cost of construction. This paper uses the shadow engineering method to evaluate the value of the runoff regulation function. The evaluation formula as follows:

(6) $$\begin{array}{c} V_{3}=Q_{\max}\times Ci. \end{array}$$

In the formula, *V*_3_ is the functional value of wetland regulation of runoff services; *Q*_max_ is the maximum safe flood regulation and storage capacity; *Ci* is the cost of building a reservoir per cubic meter of storage capacity.

The article "Big Data Technology Oriented to Wetland Resource Ecosystem Value Evaluation" was published in 2022. Journal: Comput Intell Neurosci.

## 3. Case Analysis

The original data of this case includes coastal wetland distribution data from the wetland resource survey, questionnaire survey and expert consultation data, natural characteristics of coastal wetlands, environmental statistics, socioeconomic, meteorological and hydrological data, statistical yearbooks of coastal provinces and documentary evaluation cases of typical coastal wetlands in China. To avoid repetitive calculation problems, based on previous classifications, the coastal wetland ecosystem services are divided into two parts: intermediate services and final services, regard the final service as the ecosystem service function of China's coastal wetlands, including material production, flood regulation and storage, carbon sequestration, atmospheric regulation, climate regulation, wave elimination and shore protection, land promotion, and leisure tourism. On this basis, through beneficiary analysis to determine the local, beneficiaries at three levels: provincial, national, and global [16], build a hierarchical model of dimensional analysis. In order to quantify the quantitative relationship between services, through questionnaire surveys and expert consultation data, investigate the importance of ecosystem services among beneficiaries at different levels, use the analytic hierarchy process to conduct multilevel analysis of the survey results, obtain the dominant service functions of different levels of coastal wetland ecosystem service functions, and calculate the comprehensive weight of the coastal wetland service value, as listed in Table 3.

The article "Big Data Technology Oriented to Wetland Resource Ecosystem Value Evaluation" was published in 2022. Journal: Comput Intell Neurosci.

On these basis select 62 typical coastal wetland assessment cases, covering Liaoning, Hebei, Shandong, Jiangsu, Shanghai, Zhejiang, Fujian, Guangdong, Guangxi, Hainan, and other provinces along the coast of China, extract 349 coastal wetland ecosystem service value evaluation data through data analysis, use the consumer price index to uniformly adjust the value observations in different evaluation base years to the 2013 price level of the wetland resource survey, common service types, and evaluation method types are unified as model variables. The value of 0 or 1 is used to characterize the service type and evaluation method corresponding to the evaluation data. The values of all other variables in the model are obtained by analyzing and calculating collected wetland distribution, wetland nature, environment, socioeconomic data, statistical yearbooks, etc. Based on this, a coupled evaluation model of coastal wetland ecosystem services in the form of formula (2) is constructed, and carry out the model least square parameter calibration and accuracy verification, and calculate the coefficients of the regression model for the value of coastal wetlands in China [17]. Coupled evaluation using the spatial analysis model with the regression model coefficients to obtain the coupled analysis model of China's coastal wetland ecosystem services big data, it is used to evaluate the ecosystem service value of coastal wetlands. In the process of model construction, outliers were eliminated by the 2.5 times standard of standardized residuals.

### 3.1. Result Analysis

This research uses ArcGIS 10.2 software to calculate and analyze wetland-related spatial data and uses SPSS 17.0 software for statistical data analysis. After completing the data processing, perform the leave-one-least-squares cross-checking and solving of the model and apply the model to the evaluation of the ecosystem service value of coastal wetlands in China [18]. To obtain food production, raw material production, flood regulation, water conservation, and water conservation of China's coastal wetlands, the value per unit area and total value of water purification, wave elimination, bank protection, land promotion, carbon sequestration, atmospheric regulation, leisure tourism, etc, are to be analyzed (Figure 1). Through the evaluation results, it can be known that, the service value of China's coastal wetland ecosystems, from high to low, are water conservation, water purification, food production, leisure tourism, wave elimination and bank protection, siltation promotion, land creation, flood regulation, raw material production, carbon sequestration, atmospheric regulation. The total value of coastal wetland ecosystem services obtained through the accumulation of service values is 5010.32 × 108 yuan/year. On the whole, the ecosystem service value of coastal wetlands and lakes and marshes in China are relatively close. However, due to different evaluation methods, there is a nearly fourfold difference in the evaluation results.

The article "Big Data Technology Oriented to Wetland Resource Ecosystem Value Evaluation" was published in 2022. Journal: Comput Intell Neurosci.

On the whole, the wetland ecosystem service value evaluation method based on big data proposed in this study starts from the mechanism of wetland ecosystem service value, on the basis of determining the quantitative relationship between service functions, studying the supply relationship between coastal wetlands and ecosystem services through spatial analysis, and defining the general paradigm of wetland ecosystem service value evaluation from the perspective of space and attributes, coupled with multisource wetland feature data through mathematical models to achieve quantitative evaluation of the value of wetland ecosystem services. The method verification was carried out with the evaluation of coastal wetland value as a case, and it shows that the big data analysis method can be applied to the evaluation of the service value of the wetland ecosystem [2, 19]. Through the case study, it can be found that, compared with traditional wetland ecosystem service value evaluation methods, the evaluation method based on big data has the following characteristics: (1) Based on the mechanism of wetland ecosystem services, determine services and weights through dimensional analysis so that the evaluation process has a good theoretical basis, avoid the blindness of the value evaluation process, greatly reduce repetitive calculations. (2) Big data analysis methods couple various data that affect the value of wetland ecosystem services, and through the typical wetland evaluation case for model verification and solution, to ensure the objectivity of the evaluation process, all service values are weighted manually. The final value is calculated from the real data of the wetland, the combination of objective data and cognitive knowledge is realized, and the reliability of evaluation theory and the objectivity of evaluation data are guaranteed.

## 4. Conclusion

The types of wetland ecosystems are diverse and very complex. Wetland ecosystem services have the characteristics of temporal and spatial heterogeneity, scale effect, complex mechanism, and difficult to accurately measure. Traditional methods provide scientific and feasible technical means for the observation and assessment of wetland ecosystem services. The evaluation of the service value of a single ecosystem based on the wetland case is relatively mature; however, scientific assessment of large-scale wetland ecosystem services still faces challenges. It is manifested in many aspects such as continuous observation and evaluation of time and space, definition of service quality and quantity, multiscale collaborative research, and scientific accurate measurement. With the development of information technology, wetland observation network and remote sensing Earth observation have given birth to big data on wetland ecology. The Wetland Ecosystem Observation Network will assess the moisture, long-term networked observations of soil, atmospheric environment elements, and organisms, obtain dynamic and long-term wetland ecological parameter data. Earth observation by remote sensing can realize the integration of space, space, and ground wetland observation. The combination of the two will help build a big data observation system for China's wetland ecology. It provides new opportunities for the research on complex issues of wetland ecosystem service value evaluation. Wetland ecosystem service value evaluation method based on big data, through comprehensive observational data help to solve the limitations of traditional case point evaluation methods. Therefore, it is suitable for large-scale wetlands with similar types, such as coastal wetlands, lake wetlands, river wetlands. However, the assessment methods and conditions of various types of wetlands are too different. The feasibility of the method needs to be further studied. Through wetland observation big data for global coupling modeling, solve the problem of geographical heterogeneity to a large extent. This method has good regional applicability and can solve the problem of extrapolating the value of wetland ecosystem services in different regions.

The article "Big Data Technology Oriented to Wetland Resource Ecosystem Value Evaluation" was published in 2022. Journal: Comput Intell Neurosci.

## Figures and Tables

**Figure 1:** Service value evaluation.

**Table 1:** Wetland types and ecosystem service supply matrix.

In the class	Supply service			Regulating services		
	The raw materials	Aquatic products	The water supply	The atmosphere to adjust	The water quality purification	Bio-productivity
The river	*N*	*N*	*N*	*N*	*N*	*N*
Pits or	*N*	*N*	*N*	*N*	*N*	*N*
Yantian	*N*	*N*	*N*	*N*	*N*	*N*
Culture zones	*N*	*N*	*N*	*N*	*N*	*N*
Sandy beaches	*N*	*N*	*N*	*N*	*N*	*N*
Muddy tidal flats	*N*	*N*	*N*	*N*	*N*	*N*

**Table 2:** Common attribute indicators of wetland ecosystem service value evaluation.

Project	Index content
Natural indicators	Wetland area, type, patch number, patch density, shape index, etc.
Environmental indicators	Wetland topography (altitude, slope), climate (air temperature, accumulated temperature, precipitation), etc.
Socioeconomic indicators	Population, population density, economic development, industrial, and agricultural production, etc.

**Table 3:** The relative comprehensive weight of coastal wetland ecosystem service functions.

Coastal wetland service function	The weight	Coastal wetland service function	The weight
Food production	0.1344	Wave revetment	0.1296
Raw material production	0.1037	Promote silting epeirogenic	0.0593
Bioproductivity	0.068	Carbon sequestration	0.0481
Water conservation	0.1255	The atmosphere to adjust	0.0910
The water quality purification	0.1185	Leisure travel	0.1210

## Data Availability

The data used to support the findings of this study are available from the corresponding author upon request.

## References

[1] Sannigrahi S., Chakraborti S., Joshi P. K. (2019). Ecosystem service value assessment of a natural reserve region for strengthening protection and conservation. *Journal of Environmental Management*.

[2] Sun T., Lin W., Chen G., Guo P., Zeng Y. (2016). Wetland ecosystem health assessment through integrating remote sensing and inventory data with an assessment model for the hangzhou bay, China. *The Science of the Total Environment*.

[3] Payakachat N., Tilford J. M., Ungar W. J. (2016). National database for autism research (ndar): big data opportunities for health services research and health technology assessment. *PharmacoEconomics*.

[4] Kirubakaran B., Ilangkumaran M. (2016). Selection of optimum maintenance strategy based on FAHP integrated with GRA-TOPSIS. *Annals of Operations Research*.

[5] Sahoo B., Bhaskaran P. K. (2016). Assessment on historical cyclone tracks in the bay of bengal, east coast of India. *International Journal of Climatology*.

[6] Fu S., Gao J., Zhao L. (2020). Integrated resource management for terrestrial-satellite systems. *IEEE Transactions on Vehicular Technology*.

[7] Burlakova L. E., Hinchey E. K., Karatayev A. Y., Rudstam L. G. (2018). U.s. epa great lakes national program office monitoring of the laurentian great lakes: insights from 40 years of data collection. *Journal of Great Lakes Research*.

[8] Vinten A., Kuhfuss L., Shortall O., Stockan J., Ibiyemi A., Mayc L. (2019). Water for all: towards an integrated approach to wetland conservation and flood risk reduction in a lowland catchment in scotland. *Journal of Environmental Management*.

[9] Chowdhury A., Maiti S. K. (2016). Identification of metal tolerant plant species in mangrove ecosystem by using community study and multivariate analysis: a case study from indian sunderban. *Environmental Earth Sciences*.

[10] Chen J., Wang C., Shen Z.-J., Gao G.-F., Zheng H.-L. (2017). Insight into the long-term effect of mangrove species on removal of polybrominated diphenyl ethers (pbdes) from bde-47 contaminated sediments. *The Science of the Total Environment*.

The article "Big Data Technology Oriented to Wetland Resource Ecosystem Value Evaluation" was published in 2022. Journal: Comput Intell Neurosci.

[11] Alminagorta O., Rosenberg D. E., Kettenring K. M. (2016). Systems modeling to improve the hydro-ecological performance of diked wetlands. *Water Resources Research*.

[12] Fang L. L., Valverde-Pérez B., Damgaard A., Plósz B. G., Rygaard M. (2016). Life cycle assessment as development and decision support tool for wastewater resource recovery technology. *Water Research*.

[13] Cleland J., Hutchinson C., Mcbain C. (2021). Developing dimensions for a new preference-based quality of life instrument for older people receiving aged care services in the community. *Quality of Life Research*.

[14] Bhangare R. C., Ajmal P. Y., Rathod T. D., Tiwari M., Sahu S. K. (2019). Experimental and theoretical determination of henry’s law constant for polychlorinated biphenyls: its dependence on solubility and degree of chlorination. *Archives of Environmental Contamination and Toxicology*.

[15] Yang Y., Chen T. (2019). Analysis and visualization implementation of medical big data resource sharing mechanism based on deep learning. *IEEE Access Analysis and Visualization Implementation of Medical Big Data Resource Sharing Mechanism Based on Deep Learning*.

[16] Zhang G. (2016). Research on the applications of big data on artistic designing and its influences on the design behavior. *International Journal of Technology Management*.

[17] Benedict S. H., El Naqa I., Klein E. E. (2016). Introduction to big data in radiation oncology: exploring opportunities for research, quality assessment, and clinical care. *International Journal of Radiation Oncology, Biology, Physics*.

[18] Zhang B., Tian H., Lu C. (2017). Methane emissions from global wetlands: an assessment of the uncertainty associated with various wetland extent data sets. *Atmospheric Environment*.

[19] Rebelo A. J., Morris C., Meire P., Esler K. J. (2019). Ecosystem services provided by South African palmiet wetlands: a case for investment in strategic water source areas. *Ecological Indicators*.

